# The Heuristic Algorithm Optimization of Home Care Path Based on the Internet of Things Realizes Connected Medical Care

This article has been retracted.

**DOI:** 10.1155/2022/3237554

**Published:** 2022-02-15

**Authors:** Jinfeng Zhang, Xin Li, Yu Zhao

**Affiliations:** ^1^Jilin Engineering Vocational College, Siping 136001, China; ^2^Zhejiang University, Hangzhou 310063, China

## Abstract

Optimize the scheduling problem of family nursing staff according to the actual needs of the customers, combined with the psychological behavior characteristics of the participants, and use the path heuristic algorithm on home nursing service institutions, full-time nursing staff, and nursing customers. Taking this as the maximization of the three subjects as the ultimate goal of home caregiver optimization and scheduling, a path heuristic-based heuristic optimization and scheduling method (path heuristic algorithm, PHA). The effectiveness of this method is analyzed through examples, and finally, according to the experimental analysis results of the distribution, dominance, and convergence of the proposed PHA algorithm, the home caregiver optimization and scheduling method proposed in this paper can provide a more long-term scheduling method for enterprise companies.

## 1. Introduction

Family medical and nursing services mainly refer to the provision of hospitals, communities, rehabilitation care, and basic life services as the main body, according to their specific personnel, do not need services [1–3]. This model changes the existing medical and service model, where demand users can order different types of care tasks at home without leaving out [3–5]. A difficult problem that gradually arises in the process of operation of home medical care and nursing services is the reasonable arrangement of caregivers to ensure that the task costs the least while meeting the needs of users. Today, the service standard of home medical caregivers is to provide services to users in need in community hospitals and home nursing professional companies, and finally return to their starting point. Scientific and reasonable scheduling and optimizing the user service of full-time nursing personnel are actually a full guarantee for the reasonable use of resources, which can effectively improve the user roaming ground and service quality. However, because the medical service time needs to be closely related to the physical condition of the household, in general, customers need door-to-door service time is uncertain, which will increase the difficulty to solve the optimization and scheduling problems of family nursing staff [6–9].

According to the above analysis, the current research on the older customer demand optimization and electroplating research, considering the customer will face emergency losses, will bring potential risks, according to previous research results from customer needs, nursing staff, and home nursing institutions; these three aspects, in the process of solving algorithm, proposed path heuristic algorithm can be effective for the family medical staff scheduling optimization method support.

## 2. Problem Description and Model Building

### 2.1. Problem Description

The family nursing staff scheduling problem studied in this paper is described as follows: home nursing institutions have K nursing staff, need to serve the elderly customers in different locations, during the service process, each caregiver starts from the agency, follow the planned route to the designated customer, then return to the institutional center; each caregiver can serve multiple elderly clients, but each elderly customer can only be served by one caregiver; each customer has its own time window to receive the service, if the caregiver pays the waiting costs in advance, late to bear the operating costs, nursing staff skill level meets customer needs; in this case, with the minimum total operating cost of the nursing center, get an initial caregiver scheduling with a path optimization scheme.

When the nursing staff performs the service according to the initial scheduling plan, there are three kinds of optimization events: customer temporary change time window, new emergency demand, and temporary cancellation in the system, which makes it difficult to implement the original initial scheduling plan. In this case, based on the optimization of the system state, the effective optimization and scheduling model are studied and quickly formulate the adjustment scheme to minimize the perturbation to the original scheme [10–12].

To facilitate the construction of the model, the following assumptions are made on the above questions:

1. The initial plan of nursing staff dispatch is known
2. After the optimization occurs, the customers who are being served by the home care staff are regarded as completed customers
3. The position of each nursing staff during optimization is a virtual nursing center, which is the starting point of service after disturbance, and the initial home care center is the end of service
4. As the nursing staff resources of the institution are limited, when formulating the adjustment plan, it is assumed that the remaining tasks are completed by the nursing staff of the initial plan

### 2.2. Mathematical Model

The problem studied in this paper can be defined on a connected graph *G* = (*V*, *A*), where *V* = {0, 1, 2, ⋯, *n*} is a set of points, and an arc set. *A* = {(*i*, *j*)|*i*, *j* ∈ *V*, *i* ≠ *j*} Point 0 indicates the home care center or office, and other points {1, 2, ⋯, *n*} indicate the location of the customer. *i* ∈ *Ns*_*i*_[*e*_*i*_, *l*_*i*_]*e*_*i*_*l*_*i*_*s*_0_ = *s*_*n*+1_ = 0*e*_*n*+1_ = *e*_0_*l*_*n*+1_ = *l*_0_*i* ∈ *Nd*_*i*_ ∈ *Dk* ∈ *Kr*_*k*_ ∈ *Di* ∈ *Nk* ∈ *Kd*_*i*_ ≤ *r*_*k*_. For demand, the service duration is, and the service must be performed within the time window, which cannot start immediately before arrival and later than arrival. For home care companies, for the earliest time for all caregivers to start work, for the latest time for all caregivers to return to the company. Make the set of capability levels specified by the company D. Yes, it indicates the level requirements for the requirement *i*. Make K a collection of all of its caregivers. Yes, it represents the service level of nursing staff Cang. All services need to meet the principle of grade matching, yes, and, at the time, caregiver k to service requirements *i*. The total cost of the problem includes the fixed cost of the caregivers, the cost of service and on route. For nursing staff, the fixed cost of daily service is, the service cost of customer *i* is, and the travel cost is numerically equal to the travel time. *k* ∈ *Kf*_*k*_*v*_*k*_*s*_*i*_.

Based on the above description and the mathematical notation, the mathematical model of the problem is as follows:

(1) $$\begin{array}{c} \mathrm{Minimize}\underset{k\in K}{\sum }\underset{j\in N}{\sum }f_{k}x_{0jk}+\underset{k\in K}{\sum }\underset{i\in V}{\sum }\underset{j\in V}{\sum }v_{k}s_{i}x_{ijk}+\underset{k\in K}{\sum }\underset{i\in V}{\sum }\underset{j\in V}{\sum }t_{ij}x_{ijk}, \end{array}$$

(2) $$\begin{array}{c} \text{Subject to }\underset{j\in V}{\sum }x_{0jk}=1\;\forall k\in K, \end{array}$$

(3) $$\begin{array}{c} \;\underset{j\in V}{\sum }x_{ijk}-\underset{i\in V}{\sum }x_{jik}=0,\;j\in \frac{V}{\left\{0\right\}},k\in K, \end{array}$$

(4) $$\begin{array}{c} \underset{i\in V}{\sum }x_{i,n+1,k}=1\;\forall k\in K, \end{array}$$

(5) $$\begin{array}{c} \underset{k\in K}{\sum }\underset{j\in V}{\sum }x_{ijk}=1\;\forall i\in N, \end{array}$$

(6) $$\begin{array}{c} e_{i}\leq T_{i}\leq l_{i}\;\forall i\in V, \end{array}$$

(7) $$\begin{array}{c} T_{i}+s_{i}+t_{ij}-T_{j}\leq M\times \left(1-x_{ijk}\right),\forall i,j\in V,\forall k\in K, \end{array}$$

(8) $$\begin{array}{c} T_{i}=T_{j},\forall \left(i,j\right)\in P, \end{array}$$

(9) $$\begin{array}{c} x_{ijk}\in \left\{0,1\right\},\forall i,j\in V,\forall k\in K. \end{array}$$

The objective function (1) represents minimizing travel costs and customer demand costs. The constraint (2) indicates that each customer can only be served once. Constraint (3 ~ 5) indicates that each service person starts from the starting point 0 and returns to the starting point after serving several customer points. Constraints indicate that no child loop exists in the path. Constraints indicate that the total demand of paramedics to serve customers cannot exceed the maximum service capacity. The equation is a computational expression for the cost of the customer demand. Constraints (9) indicates the decision variable is 0-1 variable.

## 3. Solution Method of the Optimization and Scheduling Model

The scheduling optimization and scheduling problem of family caregiver studied in this paper are a multiobjective combination optimization problem, which belongs to the NP-hard problem and is difficult to solve with an accurate algorithm and needs to design an efficient group intelligent optimization algorithm. A new group intelligent optimization algorithm proposed in 2016 has the characteristics of few artificial setting parameters, fast convergence speed, and easy implementation, which has been applied in many fields, but the algorithm also has defects of local optimal, premature convergence, and not high solving accuracy. To this end, we propose an improved path heuristic algorithm for the optimization and scheduling problems.

### 3.1. Encoding and Decoding

The problem studied in this paper involves two subproblems of nursing staff assignment and senior customer service ranking. For this kind of problems, the two-stage coding method is generally adopted. However, as the number of customer points increases, this method will increase the dimensionality of the individual whale groups, causing the algorithm to slow down. In this paper, *X* = {*X*_1_, *X*_2_, ⋯, *X*_*N*_} is used to represent the position of a whale group. *N* is the number of customers, where *X*_1_, ⋯, *X*_*N*_ is the random number generated between (1, *D* + 1), and *D* is the number of medical staff. The integer part is the nursing staff assigned by the customer, and the size of the decimal part determines the order of customer service. Based on random key descending encoding method rearranges the decimal part, after arrangement: the position of the component corresponds to the customer's service order. Take 6 customers requiring 3 caregiver on-site service as an example to illustrate the encoding and decoding of a group of whales. The position of a group of whales is *X* = [3.238, 1.334, 3.945, 2.128, 1.637, 2.239], the decoding process is shown in Figure 1. From Figure 1, we can see that customer 1, customer 2, customer 3, customer, 1, customer 5, and customer 6 assigned care. The personnel are 3, 2, 1, 3, 1, and 2. Sort the decimals of the components in descending order to get the customer service order is 3, 5, 2, 6, 1, 4. The arrangement is 5-2; the service arrangement of nursing staff 2 is 6-4, and the service arrangement of nursing staff 3 is 3-1.

### 3.2. Chaos Initializes the Population

The initialized population of the standard WOA algorithm is generally generated at random and does not guarantee the uniformity of the solution distribution in the search space. Chaos sequence has the characteristics of randomness, ergodic nature, regularity, etc. Population initialization can ensure population diversity and uniformity. The literature has verified that tent maps perform better than logistic maps in ergodic uniformity. Therefore, in this paper, the mathematical model of tent chaotic map initializing the tent chaotic map is as follows:

(10) $$\begin{array}{c} y_{k+1}=\left\{\begin{array}{c} 2y_{k},0\leq y_{k}<0.5,\\ 2\left(1-y_{k}\right),0.5\leq y_{k}\leq 1. \end{array}\right. \end{array}$$

The steps to initialize the population based on tent chaotic mapping are as follows:

**Step 1 .**

First, take *D* random numbers *y*_*d*1_^0^, *d* = 1, 2, ⋯, *D* between (0,1), and generate a vector *y*_*i*+1_^0^ = (*y*_1,*i*+1_^0^, ⋯, *y*_*d*,*i*+1_^0^, ⋯, *y*_*D*,*i*+1_^0^) according to the tent mapping function, where each component *y*_*d*,*i*+1_^0^ is expressed as

(11) $$\begin{array}{c} y_{d,i+1}^{0}=\left\{\begin{array}{c} 2y_{di}^{n},0\leq y_{di}^{0}\leq 0.5\\ 2\left(1-y_{di}^{0}\right),0.5\leq y_{di}^{0}\leq 1 \end{array}\right.,d=1,2,\cdots ,D,i=1,2,\cdots ,n. \end{array}$$

**Step 2 .**

Map the generated chaotic variables to the decision variable space (*x*_min,*id*_, *x*_max,*id*_) to obtain the *i*-th whale position vector *X*_*i*_^0^ = {*x*_1_^0^, ⋯, *x*_*di*_^0^, ⋯, *x*_*Di*_^0^} of the initial population, where the *d*-th component *x*_*di*_^0^ is

(12) $$\begin{array}{c} x_{di}^{0}=x_{\min,id}+y_{di}^{0}\left(x_{\max,id}-x_{\min,id}\right),i=1,2,\cdots ,n;d=1,2,\cdots ,D. \end{array}$$

In the formula, *x*_max,*id*_ and *x*_min,*id*_ are, respectively, the upper and lower bounds of the search for the third dimension of the individual factory.

### 3.3. External Archive Set Update and Maintenance

In the PHA algorithm, the nondominant solution set is saved using a fixed-scale external archive set. During the cable process, the new populations are sorted by NSGA-II to find noninferior solution sets [13, 14]. Each individual in the new nonpoor solution set was updated to the external archive set. If the updated external file size exceeds the set maximum value. Archives require pruning and maintenance. Relevant scholars demonstrate that the 3-point shortest path method has advantages in maintaining population distribution and diversity. Therefore, this paper uses this method for pruning.

### 3.4. The Convergence Factor Is Nonlinear Adjustment Strategy

The convergence factor *α* in the standard WOA algorithm decreases linearly from 2 to 0 throughout the iteration. This linear decreasing strategy easily makes the algorithm trapped locally optimally. In this paper, we introduce nonlinear-varying cosine functions to improve the convergence factors.

(13) $$\begin{array}{c} \alpha =\alpha_{\text{initial}}+\left(\alpha_{\text{initial}}-\alpha_{\text{final}}\right)\left(\frac{1-\cos\pi l/t_{\max}}{2}\right). \end{array}$$

Among them, *α*_initial_ and *α*_final_ are the maximum and minimum values of the convergence factor *α*, and *t* is the current iteration number of the whale group. *t*_max_ is the maximum number of iterations.

This improvement strategy has slow convergence factor in the early iteration, which helps the whale to find the optimal solution with a large step length, makes the algorithm has strong global search ability, the stable change rate decay of the convergence factor ear in the later stage, and facilitates the local search in the late search to find the optimal solution. This can well balance the global exploration and local search ability of the algorithm.

### 3.5. Change the Neighborhood Search Policy

#### 3.5.1. Insert

The structure is constructed by randomly selecting any customer point on the selected path except the distribution center point and inserting the customer into all the other possible locations except in the original location. As shown in Figure 2, customer 2 is moved between customer 3 and customer 4 on this path.

#### 3.5.2. Inverse Order

The structure is to select any two locations from the current feasible path to arrange the two customers in reverse order. As shown in Figure 3, customer 1 and customer 5 are inverted on that path.

### 3.6. Algorithm Process

**Step 3 .**

Basic parameters of the initialization algorithm: set the maximum number of iteration of *N*′, the number of dimension *D*, helical shape constant *b*, convergence factor *α*, and neighborhood search; chaotic initialize the population. *t*_max_.

**Step 4 .**

Convert the individual position of each whale member in the population to the service path of each caregiver according to the coding and decoding rules. The corresponding three subtarget values were also calculated, and the initial population was sorted using the fast nondominant ranking and crowding distance of NGSA-II, and the first *N*′ elite individuals were selected to deposit into the external archive set.

**Step 5 .**

If *t* < *t*_max_, update *α*, *A*, *C*, *l*, and *p*, when *q* < 0.5, if ∣*A* | ≥1, randomly select a whale individual position *X*_rand_ in the current population, and update the current whale by formula (14) position; if ∣*A* | <1, determine the position of the whale by formula (15). When *p* ≥ 0.5, update the individual position of the whale by formula (16).

(14) $$\begin{array}{c} X\left(t+1\right)=X_{\mathrm{rand}}\left(t\right)-A\cdot \left|C\cdot X_{\mathrm{rand}}\left(t\right)-X\left(t\right)\right|, \end{array}$$

(15) $$\begin{array}{c} X\left(t+1\right)=X_{p}\left(t\right)-A\cdot \left|C\cdot X_{p}\left(t\right)-X\left(t\right)\right|, \end{array}$$

(16) $$\begin{array}{c} X\left(t+1\right)=D^{t}\cdot e^{bl}\cdot \cos\left(2\pi l\right)+X_{p}\left(t\right). \end{array}$$

Among them, *X*_*p*_ is the position of the prey. Since the noninferior solution set in the current population is stored in the external file, one is randomly selected from the noninferior solution set as the position of the prey.

The updated whale populations were merged with contemporary population evolution to generate new populations, used the fast nondominant ranking method and crowded distance to find the noninferior solution set, and to update and maintain external files.

**Step 6 .**

10% of individuals are randomly selected from the external file for the variable field search. If the obtained new solution can dominate the original solution, it is used instead; otherwise, the original solution is retained.

**Step 7 .**

To determine whether the termination condition is reached, yes, the service path and target function value of each caregiver are output to terminate the algorithm, otherwise, go to step 4.

### 3.7. Analyses of Simulation Experiments

In order to verify the effectiveness of the PHA algorithm, this paper compares the PHA algorithm with the MOWOA algorithm and the NSGA-II algorithm. The algorithm parameters in this paper are set as upper spiral shape constant *b* = 1, initial value of convergence factor *α*_initial_ = 2, end value of convergence factor *α*_final_ = 0, population size and external archive size are both 60, the number of variable neighborhood searches is 30, and the maximum iteration number is 100.

### 3.8. Example Description

Since there is no standard test dataset for the optimization and scheduling problems of home caregiver scheduling, two classes of cases are adopted in the paper to verify the effectiveness of the PHA algorithm. One is based on the typical Solomon test case cut, random selection of C103, R103, R202, and RC108 cases in the test question library for testing. With only customer-specific parameters in these examples, no parameters related to caregiver costs were involved. Therefore, according to the problems studied in this paper, the unit service cost of nursing staff cost, late operation cost, early arrival cost, and unit distance travel cost is reasonably added, which are 250, 18, 15, and 3, respectively. The other category is random generation examples, described as follows: elderly customers are evenly dispersed in the two-dimensional plane [0,100]^2^. The home care center is located at point (50,50), where the nursing staff journey time is measured by Euclidean distance, and the customer service time is evenly distributed to *U* [15,30]. The time window is calibrated by the randomly generated center and width. For client *i*, the time window center cen_*i*_ is the interval (*e*_0_ + *t*_0*i*_, *l*_0_ − *t*_0*i*_ − *s*_*i*_), where *e*_0_ = 0, *l*_0_ = 600, and *t*_0*i*_ are the time from the care center to the client *i*. *s*_*i*_ is the customer's service time, the time window width *w*_*i*_ of customer *i* is a random integer between *U* [50,90] uniformly distributed, the time window of customer *i* is [*e*_*i*_, *l*_*i*_] = [cen_*i*_ − 1/2*w*_*i*_, cen_*i*_ + 1/2*w*_*i*_], and the parameters of the nursing staff related cost are the same as the first type of case.

According to the data in the randomly generated example, the standard whale swarm algorithm is used to obtain a satisfactory initial delivery plan with the goal of the lowest total service cost: the service path of nursing staff 1 is 0-14-21-26-30-11-13-0; the service path of nursing staff 2 is 0-15-2516-23-11-6-0; the service path of nursing staff 3 is 0-10-5-2-18-9-17-0; the service path of nursing staff 4 is 0-24-22-25-7-23-3-0; the service path of nursing staff 5 is 0-14-5-24-29-3-8. The service path of the caregiver in the initial solution is shown in Figure 4.

At the original plan execution time *T* = 50, the following three optimization events occurred: a new customer demand with coordinates of (50,20), the time window is [63,73], the time window of customer 3 was changed from [115,125] to [106,116], and customer 11 cancelled the service due to temporary problems. Discovered by analysis, older customers are more sensitive to earnings and losses than their nursing facilities and caregivers. Order *α*_1_ = *β*_1_ = 0.92, *λ*_1_ = 3.5; *α*_2_ = *β*_2_ = 0.88, *α*_3_ = *β*_3_ = 0.88, *λ*_2_ = *λ*_3_ = 2.25, *γ* = 0.61, and *δ* = 0.69. Assuming that the subjective probability functions for the three demand changes are [*p*_1_^*L*^, *p*_1_^*U*^] = [20%, 40%], [*p*_2_^*L*^, *p*_2_^*U*^] = [15%, 25%], and [*p*_3_^*L*^, *p*_3_^*U*^] = [5%, 10%].

### 3.9. Algorithm Performance Analysis

The evaluation index selected two indexes: uniform distribution index SP and dominance index CM. Since the true optimal Pareto leading edge of the sought problem is unknown, the set of noninferior solutions obtained by all three algorithms is approximated as the optimal Pareto cutting edge. Algorithms were tested with four standard cases and one random case, and three contrast algorithms were run 20 times for each case and obtained the mean of the SP, CM metric as shown in Table 1.

It can be seen from Table 1 that for the SP index, the SP index of PHA is better than the other two algorithms for all cases, so that the distribution of noninferior solutions on the Pareto leading edge of PHA is relatively uniform. For the CM metrics, for all cases, C (PHA − MOWOA) M O W O A) > C (MOWOA − PHA) and C (PHA − NSGA − II) > C (NSGA − 11 − PHA), indicating that the vast majority of noninferior solutions obtained by the PHA algorithm were superior compared to the other two algorithms. For example, in the R105 test problem, about 65% of the nondominant solutions of NSGA-II are dominated by PHA, while only 16% are obtained by the PHA algorithm, about 82% by PHA, and 35% are obtained by the PHA algorithm, further indicating that the improvement algorithm achieves good quality and has good search ability.

The mean can only compare the algorithm performance from the macro level. In order to further analyze the performance of the algorithm from the microlevel, the Wilcoxon signed-rank test method is used to analyze the sample data of the indicators, and the significant difference between the two algorithms is judged according to the results. For the SP and CM metrics of test cases, versus MOWOA and NGSGA-II algorithms, the PHA test results are shown in Table 2. Sig (*p* < 0.05) as Y indicates that PHA is significant relative to other algorithms.

From the table, for the SP and CM metrics, for all test issues, C (1mowo a-mowo a) is the optimal algorithm. The boxplot of the SP evaluation metrics in Figure 5 more intuitively indicates that the PHA algorithm is significant. The performance of the algorithm is also illustrated again by analyzing the four standard case Pareto fronts. Due to the limited space, only the Pareto fronts obtained from the three algorithms for the RC108 calculation examples are listed, as shown in Figure 6. It is known from the 2-D projection diagram of the solution distribution of Pareto that most of the noninferior solutions obtained by the PHA algorithm focus on the upper right of the coordinate system and mostly dominate the corresponding solutions obtained by other algorithms, which fully illustrates the good solution effect of the algorithm proposed in this paper. In summary, the PHA method designed in this paper can effectively solve the optimization problem of family care resource scheduling.

### 3.10. Effect Analysis of Optimization and Scheduling

To verify the effectiveness of the optimization and scheduling strategies, the random case is simulated, and the results are compared with the resurgent method, as shown in Figure 7. In the figure, RS is the scheme obtained from rescheduling (rescheduling) for new and old customers with minimum total scheduling cost. As seen from the two-dimensional distribution diagram of Figure 7, the solutions obtained using optimization and scheduling methods account mostly in the dominant rescheduling scheme (RS) in the satisfaction indicators of the customer and caregivers, but not in the satisfaction of the care center. This shows that the behavioral optimization and scheduling model improve the customer and nursing satisfaction based on the increased total cost of nursing facility scheduling compared to the rescheduling model. For nursing facilities, although some interests are lost in the short term, but from the perspective of long-term development, it will help enterprises to establish a good image in the industry, expand their own influence, and improve the competitiveness of the industry.

## 4. Conclusions

This paper makes daily work schedule and scheduling for different levels of home caregivers according to the different needs of customer service. We can apply the path heuristic algorithm to solve the problem and ensure that the optimal result needs to be solved, which is of great significance for practical cases. Finally, through the analysis of the experimental results, the method design used in this paper is relatively scientific and reasonable, which can effectively improve the operation volume, is significantly better than the existing charging commercial software, and provides a reference for the subsequent personnel scheduling problem.

## Figures and Tables

**Figure 1:** Individual decoding process for whales.

**Figure 2:** Path interpolin operation.

**Figure 3:** Inverse-sequential operation.

**Figure 4:** Initial scheduling scheme for the caregiver service path.

**Figure 5:** Presents the SP index box plots for the different algorithms used in this paper.

**Figure 6:** RC108 case 3 algorithms Pareto frontier.

**Figure 7:** Optimization for comparison with scheduling and rescheduling policies.

**Table 1:** Comparison of algorithm results of 5 test problems.

Example	Metric		PHA	MOWOA	NSGA-11
C101	SP		0.1711	0.2113	0.3145
	CM	C(lMOWOA-NSGA-II)	0.8032	——	——
		C(PHA -WOA)	0.8133	——	——
		C(NSGA-H-PHA)	——		0.1279
		C(MOWOA-PHA)	——	0.3452	

R105		SP	0.1733	0.2290	0.3276
	CM	C(lMOWOA-NSGA-II)	0.6624	——	——
		C(1MOWO A-MOWO A)	0.8245	——	——
		C(NSGA-H-PHA)	——	——	0.1513
		C(MOWOA-IMWOA)		0.3540	——

R202		SP	0.1356	0.1833	0.2033
	CM	C(lMOWOA-NSGA-II)	0.7834	——	——
		C(1MOWO A-MOWO A)	0.8214	——	——
		C(NSGA-H-PHA)	——	——	0.1678
		C(MOWOA-PHA)	——	0.3721	——

RC108		SP	0.0723	0.0815	0.1267
	CM	C(lMOWOA-NSGA-II)	0.6623	——	——
		C(PHA -WOA)	0.7833	——	——
		C(NSGA-H-PHA)	——	——	0.1455
		C(MOWOA-PHA)	——	0.4923	——

Random optimization (random.)		SP	0.0342	0.0508	0.0565
	CM	C(lMOWOA-NSGA-II)	0.7532	——	——
		C(1MOWO A-MOWO A)	0.6926	——	——
		C(NSGA-H-PHA)	——	——	0.3144
		C(MOWOA-PHA)	——	0.5733	——

**Table 2:** Wilcoxon fits the rank test.

Test case	Evaluation indicators	Sig (*p* < 0.05)	
		WQA	NSGA-II
C101	SP	Y	Y
	C	Y	Y
R105	SP	Y	Y
	C	Y	Y
R202	SP	Y	Y
	C	Y	Y
RC108	SP	Y	Y
	C	Y	Y
This paper case	SP	Y	Y
	C	Y	Y

## Data Availability

The labeled dataset used to support the findings of this study are available from the corresponding author upon request.
